# Clinical Value of Vitamin D, Trace Elements, Glucose, and Lipid Metabolism in Diagnosis and Severity Evaluation of Psoriasis

**DOI:** 10.1155/2022/8622435

**Published:** 2022-07-14

**Authors:** Da Huang, Liangbao Su, Lihua Zhuang, Jie Wu, Jihua Zhuang

**Affiliations:** ^1^Department of Dermatology, Wujin Hospital Affiliated with Jiangsu University, Changzhou, 213000, China; ^2^The Wujin Clinical College of Xuzhou Medical University, Changzhou, 213000, China; ^3^Department of Dermatology, Anxi County Hospital of Fujian Province, Quanzhou 362499, China; ^4^Department of Dermatology, Taicang Traditional Chinese Medicine Hospital, Suzhou, 215499, China; ^5^Department of Laboratory, The First People's Hospital of Changzhou, Changzhou, 213004, China

## Abstract

**Objective:**

The levels of vitamin D, trace elements, and glucose and lipid metabolism in psoriasis were evaluated, and their value in disease diagnosis and severity evaluation was explored.

**Methods:**

In this study, the serum trace elements, blood glucose, and blood lipid indexes of 360 patients with psoriasis and 500 healthy subjects were compared and analyzed.

**Results:**

The results of 25-(OH) D3, Cu/Zn, and HDL-C in patients with psoriasis were significantly different from those in the control group. With the aggravation of the disease, Psoriasis Area and Severity Index (PASI) was positively correlated with 25-(OH) D3 and HDL-C and negatively correlated with Cu/Zn. The AUC of the three indexes for the diagnosis of psoriasis was 0.899, 0.675, and 0.848, respectively.

**Conclusion:**

There are metabolic abnormalities of 25-(OH) D3, Cu/Zn, and HDL-C in patients with psoriasis, and paying attention to these indicators is conducive to the diagnosis of disease.

## 1. Introduction

The global incidence of psoriasis is 2% ~3%, and the incidence of Asians is 0.4%. The clinical manifestations are mainly erythema and scales. The disease can be found throughout the body, especially in scalp and limb extension [1]. The clinical manifestations are mainly erythema and scales. The disease can occur throughout the body, and the scalp and limbs are more common. The clinical treatment of the disease is difficult and easy to relapse, which seriously affects the quality of life and health of patients. The research on its pathogenesis has always been the focus and difficulty of dermatology research. Many scholars believe that it is related to the imbalance of Th1/Th2 and Th17/IL-17 and the proliferation of keratinocytes. In addition, with the deepening of research, some scholars have found that vitamin deficiency or deficiency [2], trace elements [3], and glucose and lipid metabolism [4] are ubiquitous in the serum of patients with psoriasis. However, there is no comprehensive analysis of the relationship between the three and psoriasis. In this paper, we will study the correlation between these characteristics and psoriasis, which may help us to further study the pathogenesis and even provide better ideas for its treatment.

## 2. Object and Method

### 2.1. Source of Research Object

360 patients with psoriasis admitted to our department of dermatology from January 2019 to December 2020 were selected as the study group. They all met the diagnostic criteria of psoriasis: red inflammatory papules with clear boundaries were first found, and then the lesions gradually increased or fused into plaques, showing brown red color, infiltration at the base, inflammatory erythema around the lesions, and adhesion of several layers of scales on the surface. The characteristic manifestations were film phenomenon and dotted bleeding. According to the characteristics of skin lesions, the patients were divided into four types: normal type, pustule type, joint type, and red skin type. Inclusion criteria were as follows: 18~65 years old, implementation of the study with informed consent of patients and approval by the Hospital Ethics Committee. Exclusion criteria were as follows: patients received systematic treatment four weeks before admission, including hormone, Avi A, immunosuppressant and biological inhibitor treatment, severe endocrine systemic diseases, pregnant women, lactation women and diabetes, hypertension, and mental disorders. After screening, a total of 360 patients in the study group were included, including 178 males and 182 females, with an average age of (42.98 ± 12.45) years. Normal type, pustular type, joint type, and red skin type patients were 211, 20, 104, and 25 cases, respectively. In the same period, 500 healthy patients were included in the control group. The number of males and females in the group was 247 and 253, respectively, with an average age of (43.12 ± 13.08) years.

### 2.2. Method

After admission, 2.5–3.0 mL venous blood was collected from each of the two groups for detection of related indicators. Laboratory tests included serum 25-(OH) D3, sodium (Na), potassium (K), calcium (Ca), phosphorus (P), magnesium (Mg), iron (Fe), selenium (Se), copper (Cu) and zinc (Zn), total cholesterol (TC), triglyceride (TG), low-density lipoprotein cholesterol (LDL-C), high-density lipoprotein-cholesterol (HDL-C), and fasting blood glucose (FPG). The related test items were completed by the laboratory staff of our hospital, and the final test results were obtained through the database of the calculation system of the laboratory and the physical examination center of our hospital. The determination of trace elements uses the German Roche automatic biochemical analyzer (Cobas-6000) and the company's production kit, blood glucose, and blood lipid test in patients with venous blood collected using low-speed centrifuge (Anhui Jiawen JW-1046), 3000 r/min and centrifugal 10 min and serum separation using automatic biochemical analyzer (Abbott-16000) for detection. In addition, Psoriasis Area and Severity Index (PASI) was used to evaluate the severity of lesion area in patients with psoriasis. The score ranged from 0 to 72 points. The higher the score, the more serious the disease. PASI score 12 was divided into the severe group.

### 2.3. Statistical Method

We first carry out the normality test on all data, the measurement data conforming to the normal distribution are expressed as mean ± SD, and *t*-test or one-way ANOVA was used. The enumeration data were expressed as %, and chi-square test was used for comparison between groups. Pearson correlation analysis was used for correlation analysis. ROC curve was used to evaluate the detection performance of the included indicators. All data were statistically calculated based on SPSS 21, with *P* < 0.05 as statistically significant.

## 3. Results

### 3.1. Comparison of Laboratory Results between Patients and Control Group

Results of each index of psoriasis patients in the study group and healthy control group are as follows: Table 1 and Figure 1.

### 3.2. Comparison of Laboratory Results between Different Groups in Patients with Psoriasis

The average PASI score of 360 patients with psoriasis was (23.41 ± 10.22), and the number of patients in the mild, moderate, and moderate groups was 108,131, and 121, respectively. The comparison of three groups of laboratory tests showed that 25-(OH) D3, Fe, Se, and HDL-C in the moderate group were lower than those in the mild group, and Cu, TC, TG, and FPG were higher than those in the mild group (*P* < 0.05). The differences in Zn and Cu/Zn between the moderate group and the severe group were also significant, but the Zn level in the moderate group was higher, and the Cu/Zn level in the severe group was higher (*P* < 0.05). In the severe group and the mild group, the levels of Cu/Zn and FPG were higher in the former group, while those of 25-(OH) D3, Fe, Se, Zn, and Cu were higher in the latter group, and the above indexes were statistically different (*P* < 0.05). With the aggravation of the disease, 25-(OH) D3, Fe, Se, Zn, and HDL-C showed a decreasing trend, and Cu, Cu/Zn, TC, TG, and FPG showed an increasing trend, as shown in Table 2.

### 3.3. Correlation Analysis between PASI and Each Index of Patients

PASI was negatively correlated with 25-(OH) D3, Fe, Se, Zn, and HDL-C and positively correlated with Cu, Cu/Zn, TC, TG, and FPG, as shown in Table 3.

### 3.4. Multifactor Analysis of Psoriasis

With psoriasis or not as the dependent variable (yes = 1, yes = 0), and the index with *P* value less than 0.05 between the study group and the control group as the independent variable, the multifactor logistic regression was performed. It was observed that 25-(OH) D3, Cu/Zn, and HDL-C were independent influencing factors for the incidence of patients (*P* < 0.05), as shown in Table 4.

### 3.5. ROC Curve Analysis of Each Index Predicting the Incidence of Patients

The AUC parameters of 25-(OH) D3, Cu/Zn, and HDL-C in the diagnosis of psoriasis were 0.899, 0.675, and 0.848, respectively, all of which had good sensitivity. 25-(OH) D3 and Cu/Zn had good specificity, and HDL-C specificity is low, as shown in Table 5 and Figure 2.

## 4. Discussion

The etiology of psoriasis is complex. Genetics, immunity, environment, and infection are important factors in the pathogenesis of psoriasis [5]. Among them, immune system disorder is the key factor leading to psoriasis, and its operate may be contacted to the excessive production of proinflammatory factors caused by the increase in the activity of Th1, Th17, and Th22 lymphocytes. In addition, the change of trace elements in the human body is also considered as a suspicious factor for its pathogenesis [3]. In Qadim et al.'s study, serum calcium levels in 98 patients with psoriasis and 100 patients without psoriasis were compared. It was found that 37.2% of patients with psoriasis had hypocalcemia, while the probability of hypocalcemia in the control group was much lower than that in the psoriasis group (37.2% vs. 9.0%) [6]. Psoriasis, an important systemic inflammatory disease, may have a common pathogenesis with metabolic diseases such as diabetes, insulin resistance, obesity, and cardiovascular disease, leading to multiple complications in such patients [7].

In this study, we compared the size of serum vitamins, trace elements, and related glycolipid indicators in patients with psoriasis and healthy people and analyzed the influencing factors of psoriasis. The results may have important clinical significance for the screening and treatment of patients with psoriasis. In comparison of laboratory test results, we found that the levels of 25-(OH) D3, Mg, Fe, Se, Zn, and HDL-C in patients with psoriasis were significantly lower than those in healthy people, and the levels of Cu, Cu/Zn, TC, TG, LDL-C, and FPG were significantly increased. In addition, by comparing the indicators between groups with different disease levels, it was found that with the aggravation of the patient's condition, 25-(OH) D3, Fe, Se, Zn, and HDL-C showed a decreasing trend, and Cu, Cu/Zn, TC, TG, and FPG showed an increasing trend. The correlation analysis showed that PASI was negatively correlated with 25-(OH) D3, Fe, Se, Zn, and HDL-C and positively correlated with Cu, Cu/Zn, TC, TG, and FPG. These findings are similar to previous studies. Tajjour et al. found that the serum concentration of 25-(OH) D3 in patients with psoriasis was lower than that in healthy people with normal physical examination room. In this study, 25-(OH) D3 was negatively correlated with PASI (*r* = −0.435, *P* < 0.001), and 25-(OH) D3 in patients with severe diseases was also decidedly lower than that in patients with mild or moderate diseases [8]. Vitamin D is an immunoregulatory hormone, and the inhibitory effect of T lymphocytes activated by receptors has been confirmed in many autoimmune diseases [9]. Vitamin D can regulate the secretion of IL-10 by T cells, thereby participating in the reduction of Th2 cells and reducing inflammatory response. In addition, vitamin D has been proved to be able to regulate the differentiation of keratinocytes [10]. Although the relationship between 25-(OH) D3 and PASId were obtained in this study, there was still controversy over the correlation between them. More clinical trials were needed to ensure the accuracy of our results.

Trace elements play an important role in various reactions and metabolism in human body and play a role in immune and inflammatory reactions [3]. At present, many studies have analyzed the results of serum trace element concentration in patients with psoriasis. A case-control study by Sudhakar et al. compared the serum electrolyte concentrations of 25 patients and 25 control groups. The results showed that compared with the normal group, the Na and Na/K of the former were higher (*P* < 0.001), and K was lower (*P* < 0.001) [11]. In this study, two groups of Na and K *P* value is greater than 0.05, not obvious indigenous. Basavaraj et al. found that PASI showed lower Fe content in patients with mild and severe psoriasis compared with healthy people with normal physical examination (*P* < 0.001), and the same finding was found in this study [12]. Mohammad et al. compared the serum concentrations of Cu, Zn, and Mg in the control group matched the age and gender of 40 patients with psoriasis. They observed that Zn level was negatively correlated with the severity of psoriasis, and Cu and Mg were not correlated with it [13]. This study also found that Zn was negatively correlated with the patient's condition. The difference was that Se was also negatively correlated with the severity of psoriasis, and Cu was positively correlated with it. Similarly, Aggarwal et al. also found that Cu and Cu/Zn were closely related to the severity of psoriasis [14]. Ala et al. observed that the serum Cu level of patients was higher than that of the control group [15]. We analyzed the causes of serum trace element disorder in patients, which may be related to oxidative stress. Copper is a cofactor of many enzymes and participates in cell respiration, free radical scavenging, iron metabolism, tyrosinase metabolism, and collagen synthesis [14]. In inflammatory response and psoriasis arthritis, the mechanism of the increase in copper content is still unclear, and it is generally accepted that this change is related to the increase in copper blue protein. Shahidi-Dadras et al. found that the increase in copper blue protein in patients indicates the increased risk of myocardial infarction and cardiovascular disease in patients with psoriasis [16]. Zinc is the most abundant trace element in cells. Appropriate amounts of copper and zinc can reduce free radicals and enhance the antioxidant capacity of the body [17]. It is worth mentioning that the changes of serum copper-zinc ratio can be used as biochemical indicators of antioxidant or severity. Selenium level is closely related to immune function. Wu et al. showed that selenium content was proportional to immunoglobulin content. The lower serum selenium, the lower antioxidant, and immune function [18]. World Health Organization (WHO) recommended that adults supplement selenium (50-200 *μ*g/d) and zinc (15 mg/d) daily. Only about 49% of people in China reach or exceed the recommended amount [19]. Therefore, reasonable intake of trace element supplements is necessary for the prevention or treatment of psoriasis.

For a long time, a large number of studies have been dedicated to exploring the changes in serum lipid concentrations in patients with psoriasis. It is gratifying that a large number of studies have also confirmed that dyslipidemia is prevalent in patients with psoriasis. Markstad et al. collected 25 research papers from 1980 to 2012, covering 265512 patients with psoriasis [20]. When evaluating the relationship between psoriasis severity and blood lipids, it was found that psoriasis with serious conditions had a higher incidence of dyslipidemia. Existing science suggests that metabolic disorders of TC, TG, LDL, and HDL-C are directly linked to the risk of myocardial infarction, stroke, and severe cardiovascular disease [21]. A meta-analysis of serum lipids in patients with psoriasis showed that the serum TC, TG, and LDL concentrations in patients with psoriasis were higher than those in the normal population, while the HDL concentration in patients with psoriasis was lower than that in the normal population. Even after matching BMI, this comparison still had great differences [22]. In this study, the FPG level of psoriasis patients was significantly higher than that of healthy people, while HDL-C was lower than that of normal people. Surprisingly, Markstad et al. also had similar conclusions [23]. At the same time, through logistic regression analysis, among many factors, we proved that 25-(OH) D3, Cu/Zn, and HDL-C were powerful influencing factors for patients with psoriasis. Moreover, ROC curve analysis showed that they all had good diagnostic value, and they might be used as evaluation indexes for the therapeutic effect of patients in clinic.

Psoriasis is a chronic disease, which is affected by many factors such as inflammatory response disorder, heredity, and oxidative stress. In addition to physical pain, the disease also brings patients with mental and psychological distress, seriously affecting people's normal life and interpersonal communication. Many patients hope to obtain high effective diagnosis and treatment in the early stage of disease, but at present, the diagnosis of psoriasis mainly depends on the identification of clinical symptoms, which is not enough. We need to explore the indicators that may be effective in diagnosis from multiple dimensions. We searched PubMed, MEDLINE, EMBASE, and Cochrane databases for articles on the diagnosis and management of psoriasis and found few studies on the diagnosis of psoriasis, most of which focused on exploring the treatment of psoriasis. The diagnosis of psoriasis with 25-(OH) D3, Cu/Zn, and HDL-C as indicators is a new study, which may play an important role in clinical application. However, there is also a lack of reference for relevant data in this regard, and further research is needed in the future.

In general, vitamins, trace elements, and abnormal glucose and lipid metabolism are very common in patients with psoriasis. Therefore, vitamins, trace elements, and blood lipid levels should be regularly measured in clinical practice, especially for 25-(OH) D3, Cu/Zn, and HDL-C. In addition, fasting blood glucose should be measured at least once a year. If necessary, trace elements should be supplemented in time, lipid-lowering drugs should be used, and appropriate exercise should be maintained to effectively reduce the risk of cardiovascular diseases.

## 5. Strengths and Limitations

In this study, we found that 25-(OH) D3, Cu/Zn, and HDL-C metabolic abnormalities were common in psoriasis patients and healthy controls. They may participate in the pathogenesis of psoriasis by improving inflammatory response, producing reactive oxygen species or eliminating the inhibitory effect of the immune system. Although some scholars have previously proposed that the above indicators are related to the pathogenesis of psoriasis, the diagnosis of psoriasis has never occurred before. These indicators can be obtained from the patient's blood, which is a simple and convenient diagnostic method. There are still limitations in the study. The blood indexes of patients with various types of psoriasis are not analyzed, and further studies are needed in this regard.

## 6. Conclusions

There are metabolic abnormalities of 25-(OH) D3, Cu/Zn, and HDL-C in patients with psoriasis, and paying attention to these indicators is conducive to the diagnosis of disease.

## Figures and Tables

**Figure 1:** Comparison of laboratory results between patients and control group. (a) 25-(OH) D3 in the study group and control group. (b) Na in the study group and control group. (c) K in the study group and control group. (d) Ca in the study group and control group. (e) P in the study group and control group. (f) Mg in the study group and control group. (g) Fe in the study group and control group. (h) Se in the study group and control group. (i) Zn in the study group and control group. (j) Cu in the study group and control group. (k) Cu/Zn in the study group and control group. (l) TC in the study group and control group. (m) TG in the study group and control group. (n) LDL-C in the study group and control group. (o) HDL-C in the study group and control group. (p) FPG in the study group and control group. Note: ^∗^*P* < 0.05 compared with the study group and ^∗∗^*P* < 0.001 compared with the study group.

**Figure 2:** ROC curve of each index in diagnosis of psoriasis.

**Table 1:** Differences in laboratory test results between the two groups.

Factors	Study group (*n* = 360)	Control group (*n* = 500)	*t* value	*P* value
25-(OH) D3 (ng·mL^−1^)	26.03 ± 4.35	40.68 ± 5.13	43.980	<0.001
Na (mmol·L^−1^)	140.12 ± 10.54	140.25 ± 8.43	0.201	0.841
K (mmol·L^−1^)	4.56 ± 0.94	4.51 ± 1.67	0.513	0.608
Ca (mmol·L^−1^)	0.79 ± 0.12	0.80 ± 0.14	1.096	0.273
P (mmol·L^−1^)	1.10 ± 0.08	1.11 ± 0.06	1.725	0.085
Mg (mmol·L^−1^)	1.55 ± 0.43	1.79 ± 0.31	9.512	<0.001
Fe (mmol·L^−1^)	4.20 ± 1.07	5.12 ± 1.06	12.510	<0.001
Se (*μ*g·L^−1^)	75.52 ± 16.08	89.59 ± 28.17	8.780	<0.001
Zn (*μ*mol·L^−1^)	56.60 ± 8.23	88.04 ± 10.65	46.84	<0.001
Cu (*μ*mol·L^−1^)	16.23 ± 2.40	15.52 ± 4.01	2.995	0.003
Cu/Zn	0.25 ± 0.06	0.16 ± 0.03	28.900	<0.001
TC (mmol·L^−1^)	4.59 ± 0.38	4.26 ± 0.21	16.270	<0.001
TG (mmol·L^−1^)	1.45 ± 0.49	0.95 ± 0.11	22.060	<0.001
LDL-C (mmol·L^−1^)	2.53 ± 0.35	2.45 ± 0.09	4.892	<0.001
HDL-C (mmol·L^−1^)	1.23 ± 0.28	1.43 ± 0.15	13.510	<0.001
FPG (mmol·L^−1^)	4.95 ± 2.01	4.51 ± 0.02	4.896	<0.001

Data are presented as mean ± SD, unless otherwise indicated.

**Table 2:** Comparison of laboratory results between different groups in patients with psoriasis.

Factors	Mild group(*n* = 108)	Moderate group (*n* = 131)	Severe group(*n* = 121)	*F* value	*P* value
25-(OH) D3 (ng·mL^−1^)	27.64 ± 3.02	26.28 ± 3.03^∗^	24.79 ± 3.00^∗^^#^	25.730	<0.001
Na (mmol·L^−1^)	140.03 ± 5.39	140.61 ± 5.40	139.64 ± 5.36	2.714	0.068
K (mmol·L^−1^)	4.55 ± 1.17	4.52 ± 0.96	4.48 ± 0.25	0.185	0.831
Ca (mmol·L^−1^)	0.81 ± 0.26	0.78 ± 0.15	0.76 ± 0.06	2.423	0.090
P (mmol·L^−1^)	1.11 ± 0.08	1.10 ± 0.05	1.10 ± 0.04	1.123	0.327
Mg (mmol·L^−1^)	1.62 ± 0.21	1.59 ± 0.29	1.55 ± 0.32	1.812	0.165
Cu (mmol·L^−1^)	15.36 ± 2.30	16.42 ± 2.10^∗^	16.55 ± 2.07^∗^	10.400	<0.001
Cu/Zn	0.24 ± 0.04	0.25 ± 0.06	0.27 ± 0.03^∗^^#^	12.950	<0.001
Zn (*μ*mol·L^−1^)	60.49 ± 12.78	56.18 ± 9.51	54.06 ± 10.16^∗^^#^	10.420	<0.001
Se (*μ*g·L^−1^)	80.46 ± 9.02	74.05 ± 12.79^∗^	70.66 ± 10.08^∗^^#^	23.740	<0.001
Fe (mmol·L^−1^)	4.62 ± 1.32	4.16 ± 1.20^∗^	3.75 ± 1.91^∗^^#^	9.502	0.034
TC (mmol·L^−1^)	4.01 ± 0.23	4.09 ± 0.11^∗^	4.13 ± 0.24^∗^	10.660	<0.001
TG (mmol·L^−1^)	1.31 ± 0.18	1.39 ± 0.12^∗^	1.40 ± 0.19^∗^	10.150	<0.001
LDL-C (mmol·L^−1^)	2.35 ± 0.21	2.34 ± 0.42	2.27 ± 0.14	2.689	0.069
HDL-C (mmol·L^−1^)	1.93 ± 0.32	1.82 ± 0.44^∗^	1.75 ± 0.26^∗^	7.535	<0.001
FPG (mmol·L^−1^)	4.79 ± 0.37	4.92 ± 0.26^∗^	5.10 ± 0.35^∗^^#^	26.110	<0.001

The difference between the mild group in Table 1 was statistically significant with ^∗^*P* < 0.05. The difference between the moderate group was statistically significant with #*P* < 0.05.

**Table 3:** Relationship between PASI and indexes of patients.

Factors	PASI	
	*r*	*P*
25-(OH) D3 (ng·mL^−1^)	-0.435	<0.001
Na (mmol·L^−1^)	-0.120	0.228
K (mmol·L^−1^)	-0.264	0.165
Ca (mmol·L^−1^)	-0.175	0.246
P (mmol·L^−1^)	-0.063	0.478
Mg (mmol·L^−1^)	-0.119	0.052
Fe (mmol·L^−1^)	-0.521	<0.001
Se (*μ*g·L^−1^)	-0.368	<0.001
Cu (*μ*mol·L^−1^)	0.392	<0.001
Cu/Zn	0.314	<0.001
Zn (*μ*mol·L^−1^)	-0.334	<0.001
TC (mmol·L^−1^)	0.391	0.016
TG (mmol·L^−1^)	0.447	<0.001
LDL-C (mmol·L^−1^)	0.180	0.151
HDL-C (mmol·L^−1^)	-0.304	<0.001
FPG (mmol·L^−1^)	0.476	<0.001

**Table 4:** Multifactor analysis of psoriasis.

Variable	*B*	SE	Wald-*χ*^2^	*P* value	OR	95% CI
25-(OH) D3	2.348	0.586	16.058	<0.001	10.467	5.396-15.559
Cu/Zn	2.918	0.431	45.840	<0.001	18.506	10.343-33.114
HDL-C	1.814	0.761	5.681	0.008	6.134	3.030-10.596

**Table 5:** ROC curve parameters for predicting psoriasis.

Factors	Cut off	AUC	Youden index	Sensitivity	Specificity	*P* value	95% CI
25-(OH) D3 (ng·mL^−1^)	32.61	0.899	0.751	0.920	0.830	<0.001	0.874-0.924
Cu/Zn	0.79	0.675	0.630	0.947	0.683	<0.001	0.819-0.877
HDL-C (mmol·L^−1^)	1.22	0.848	0.324	0.926	0.398	<0.001	0.636-0.714

## Data Availability

The data used to support the findings of this study are available from the corresponding author upon request.
